# The Optimization Strategy of College Students' Ideological and Political Management under the Internet+ Environment

**DOI:** 10.1155/2022/2556976

**Published:** 2022-07-15

**Authors:** Ya Zhou

**Affiliations:** School of Marxism, Southeast University, Nanjing 211189, Jiangsu, China

## Abstract

In order to better deal with the challenges brought by the changes of the external environment to the ideological and political work of college students and better solve the problems of dogma, lack of operability, and inability to adapt to the changes of the new situation and environment, this topic proposes a student management information system based on the artificial neural network. This method strengthens the construction of the student management system, deeply interprets the connotation and practical needs of ideological and political work in colleges and universities in the new environment under the background of the “Internet+” era, and is committed to further optimizing the strategy of student ideological and political work on the basis of following the principles of innovation, human nature, openness, and ecology of ideological and political work. The results show that the construction of a more scientific student teaching management information system can provide intelligent and digital technical support for the improvement of ideological and political work efficiency and teaching quality and promote the innovative development of ideological and political work in colleges and universities. Therefore, the ideological and political work in colleges and universities should gradually overcome preaching, build new methods to measure students' achievements and ideological and political arms, actively occupy the dominant power of Internet discourse, and avoid the negative impact of the network by spreading positive energy.

## 1. Introduction

Traditional university management is often in the form of meetings, documents, and other forms, which consume a lot of human and material resources. Management via Internet has improved efficiency, and compared to offline management, management via Internet is more energy-efficient and carbon-reducing, which plays a meaningful role in environmental protection.

The 2019 National Conference on Beliefs and Work Practices in Colleges and Universities made it clear that the principles of ethics and advocacy should be adhered to, and people should be regarded important in an environment for ideological and political work, ideological work and politics in colleges and universities, understand the teaching standards of colleges and universities to the greatest extent, understand the whole process of education for all, and cultivate community skills [1]. Many colleges and universities in China have been playing an important role in cultivating producers and graduates who develop relationships in moral, intellectual, physical, aesthetic, social, and other aspects. Therefore, vocational training in colleges and universities must adhere to the correct culture [2]. Colleges and universities have always been an important foundation for growing crops and providing skills for national development and prosperity. Qualified persons with high quality not only must first know the necessary qualifications and theoretical knowledge but also have a higher level of political knowledge. Therefore, in the era of “Internet+,” the ideological and political work of colleges and universities must pay attention to the political commitment of students. Based on this principle, we must conscientiously adhere to the educational concept of keeping pace with time, and through the process of innovative design and efficient operation, strengthen the function of theoretical and political principles and good teaching level, as shown in Figure 1.

## 2. Literature Review

Li and others believe that management is a universal social practice of mankind and was first formed in the West as a systematic and independent scientific theory. The history of Western governance has been marked by three developments: the administration in the 19th and 20th centuries, the ideological behavior in the 1920s and 1930s, and modern management since the middle of the 20th century [3]. Yuan and others said that these management theories are universal and have laid a management foundation for foreign academic circles to study issues related to the management of ideological and political education in colleges and universities [4]. Lee and others believe that ideological and political education in different countries has its own particularity due to their different national conditions and has its unique theoretical basis and language expression. Most of them use the terms of “civic education,” “democratic education,” “religious education,” and “political socialization” as the expression of ideological and political education or ideological and moral education [5]. Sreelatha and others have argued that in order to achieve the goal of education and morality, however, governance is necessary. As a result, exploring its management in the study of thought and behavior in colleges and universities has become a recollection and awareness of the behavior of scientists [6]. Huang's and other theoretical studies of ideological discipline management and ethics in colleges and universities, mainly based on academic management and behavior, maintain ethics and govern staff in colleges and universities [7]. Li and others systematically expounded six management models, namely, the formal model, college model, political model, subjective model, fuzzy model, and cultural model [8]. Among them, the formal model emphasizes that colleges and universities are hierarchical systems, which should reasonably reflect the authority of managers in the organization; the college model is based on democratic principles and forms the common values of the organization through the professional authority of teachers; the political model focuses on the group activities in the organization and emphasizes the unity of individuals, groups, and organizations; Chu and others said that the subjective model emphasizes the belief and understanding of individual members in the organization and pays more attention to the realization of individual goals; the fuzzy model mainly aims at the complex and unstable situation in the organization so as to deepen the individual's understanding of the organization; the cultural model emphasizes that the individual's way of thinking and behavior and belief and value system are the core of organizational culture. The interaction between individuals or groups can promote the formation of organizational norms [9]. Turner and others said that the above six theoretical models comprehensively reflect the in-depth exploration of relevant theories by foreign scholars on the basis of criticism and development and provide a new research paradigm for exploring the management model of ideological and moral education in colleges and universities [10]. Judging by the results of research by Wang Ping and others on this issue, the problems that exist in the management culture and politics in the colleges and universities generally include the following five factors. First, the business management strategy lags behind [11]. Verma and others believe that at present, colleges and universities adopt the traditional administrative command management concept, which is lack of innovation, adhering to the concept of “social standard” in management and ignoring the subjective needs of students and lacking humanism. Second, the management content is old. In terms of target management, it is pointed out that the content of target management is lack of pertinence, the planning of target management is lack of integrity, the formulation of objectives is lack of interaction, the implementation of target management is lack of flexibility, and the subjectivity of target management is lack of logic. In terms of decision-making management, it is considered that the goal orientation of its strategic decision-making is general and lacks quantitative standards. The plan focuses on the completion of short-term tasks and lacks long-term effectiveness. The investigation and decision-making system is not standardized. The information source of work decision-making focuses on the inside, the information analysis and processing is simple and rough, and the decision feedback is lack of summary and correction. Third, the management method is backward [12]. Chen et al. believe that the current problems in the management methods of college students' ideological and political education are mainly manifested in the emphasis on administrative methods, the neglect of micromanagement, the lack of practical activities, and the lack of psychological education. Fourth, the weakness of the management team points out that the construction of the management team is still lack of overall scientific planning, the overall combat capability is not coordinated with the carrying tasks, and the overall quality and positive image need to be improved. Fifth, the management mechanism needs to be improved such as lack of scientific operation mechanism. The cultivation mechanism and guarantee mechanism of management team are not perfect. The internal communication and coordination mechanism, information mechanism, and evaluation mechanism of the management system are imperfect [13].

## 3. Student Management Information System Based on the Artificial Neural Network

### 3.1. Global Evolutionary Neural Network

#### 3.1.1. General Framework of the EPNN Evolutionary Learning System

The evolutionary learning system of the neural network consists of three interrelated parts, that is, connection right evolution learning mechanism, structure evolution mechanism, and learning rule evolution mechanism. Each part of the learning system has its dependent environment and corresponding evaluation mechanism [14].  Figure 2 shows a general block diagram of an evolutionary system.

#### 3.1.2. Description of the EPNN Evolutionary Learning Algorithm

Considering the interconnection of multiple layers on the front network, assume that *X* and *Y* represent the input and output vectors of the network, respectively, yi represent the actual output of the network, and *m*, *N*, and *n* represent the number of devices accessing the network, hidden units, and output units, respectively, I/O correlation between the entry process, hidden layer, and release process can be shown as

(1) $$\begin{array}{c} x_{j}=X_{j},\\ x_{0}=-1. \end{array}$$

The above two formulas meet 1 ≤ *j* ≤ *m*:

(2) $$\begin{array}{c} x_{i}=f\left(\sum_{j=0}^{i}w_{i,j}x_{j}\right), \end{array}$$

where *m* < *i* ≤ *m*+*N*,

(3) $$\begin{array}{c} y_{i}=f\left(\sum_{j=0}^{i}w_{i,j}x_{j}\right), \end{array}$$

where *m*+*N* < *i* ≤ *m*+*N*+*n*.

In the above formula, *W*_i, j_ represents the offset or threshold of the *i*^th^ processing unit, and then, there is the following formula

(4) $$\begin{array}{c} f\left(a_{i}\right)=\frac{1}{1+e^{-a^{i}\cdot T}}\;f\left(\cdot \right)\in \left[0,1\right]. \end{array}$$

In the above formula, *T* represents an adjustable parameter, which is used to adjust the shape of S-type action function.

For all connections to the forward network, it is assumed that *m* and *n* represent the number of devices and outputs of the network, respectively, and *N* represents the hidden numbers. The structure and weight of the network are equal to one person through direct access [15]. The length of each individual is the same, and the number of hidden units contained in the corresponding neural network can be the same or different. This is determined by the state *S* of each hidden unit in the individual representation.

The fitness of individuals is determined by the connection weight, learning performance, and structural performance of evolutionary networks, expressed as follows:

(5) $$\begin{array}{c} F_{i}=F_{i}^{S}+F_{i}^{E}, \end{array}$$

where *F*_*i*_^*S*^ represents the structural performance index of the *i*^th^ individual and *F*_*i*_^*E*^ represents the connection weight learning performance index of the *i*^th^ individual.

In the study, the network and variance are used as the learning performance evaluation of connection weight and the network structure complexity index—the number of hidden units and the number of effective connections are used as the structural evaluation—so as to determine the individual fitness [16], expressed as follows:

(6) $$\begin{array}{c} F_{i}^{E}=\text{SSE}\left(i\right)={\sum_{p=1}^{p}\sum_{j=1}^{n}\left(Y_{i}^{p}-y_{ij}^{p}\right)}^{2},\\ F_{i}^{E}=N_{i}^{HN}+N_{i}^{C}. \end{array}$$

League selection is a common strategy in the research of evolutionary optimization function based on EP. In order to ensure the structural diversity in the process of evolution, in the connection weight evolutionary learning, multitrack evolutionary selection is adopted, that is, the new individual generated by mutation only competes with its parent individual, and the one with better performance can survive [17].

In structural evolution learning, the selection rules are as follows. When the fitness performance is equal, individuals with the small structure scale are preferred; for the hidden unit addition variation, only when the structural variation improves the learning performance of weight evolution and can the new individual with better performance replace the individual with the worst performance of its parent, which indicates structural evolution; and for hidden unit deletion variation, only when the structural variation does not reduce the learning performance of weight evolution, and the new individual with better performance will replace the individual with the worst performance of its parent, which indicates structural evolution [18].

In the structural variation, when the hidden unit is added and mutated, the relevant connection weight of the newly added hidden unit is set to zero, and the relevant connection weight of the original hidden unit remains unchanged. When the hidden unit is deleted and mutated, the relevant connection weight of the original hidden unit remains unchanged. The purpose of this is to expect good performance changes between father and son generations before and after structural variation, and the generation gap should be as small as possible [19].

In EPNNA, first, evolutionary learning is carried out for the fully connected forward network, and finally, the learned network is pruned. Structural variation includes three basic operators: hidden unit addition variation, hidden unit deletion variation, and connection pruning variation.

(1) Implicit unit addition variation: after variation, the number of *i*^th^ individual hidden units in the population is

(7) $$\begin{array}{c} N_{i}^{H}\left(t+1\right)=N_{i}^{H}\left(t\right)+U\left[1,\Delta_{\max}\right], \end{array}$$

where Δ_max_ represents the maximum number of hidden units allowed to be added or deleted per structural variation, and *U*[1, Δ_max_] represents the uniformly distributed random number between 1 and Δ_max_.

(2) Hidden unit deletion variation: after variation, the number of *i*^th^ individual hidden units in the population is

(8) $$\begin{array}{c} N_{i}^{H}\left(t+1\right)=N_{i}^{H}\left(t\right)-U\left[1,\Delta_{\max}\right]\;N_{i}^{H}\left(t+1\right)\geq 1. \end{array}$$

Randomly select *N*_*i*_^*H*^(*t*+1) hidden units from the individual hidden unit queue and delete their related connections in the individual network.

### 3.2. Connection Pruning Variation

For the individual network with a satisfactory fitness value, the connection pruning variation is determined according to the number of connections whose connection weight tends to. In the prunable case, each mutation deletes one of the least important connections from the network [20].

When and only when the population evolution stagnates or a satisfactory solution is obtained, the connection weight learning is ended and the process of structural evolution learning is transferred. In the process of structural evolution learning, different structural variations are adopted according to whether a satisfactory solution is obtained [21]. When the satisfactory solution is obtained, the structure pruning mutation is carried out. For the pruned structure network population, the connection weight evolutionary learning is carried out. When the satisfactory solution is not obtained and the evolution is stagnant, the structure growth mutation is carried out. Then, the connection weight evolutionary learning is carried out for the new structure scale network population. When the structure pruning evolution stops, the evolutionary learning process is ended and the satisfactory optimal solution obtained by evolutionary learning is determined [22].

The overall evolutionary neural network process is shown in Figure 3.

The detailed steps of the algorithm are as follows.

(i) Initialize the population, as shown in the following formula:
  (9) $$\begin{array}{c} x_{t}\left(t\right)=\left[W_{t},C_{i}\right],i=1,2,\ldots ,N_{\text{POP}}\;t=0\text{ gen}S=0. \end{array}$$
(ii) The connection weight learning algorithm process is described in the following algorithm process. If the evolution stagnates or a satisfactory solution is obtained, end the connection right learning and move to the next step 3. Otherwise, continue the connection right learning process.

### 3.3. Effectiveness Analysis

For the initial structural network population, if the satisfactory solution is obtained, the structural modification variation and connection weight learning can be carried out. Otherwise, when the satisfactory solution is not obtained, the evolution of connection weight stagnates. It shows that the current population does not have the structure to obtain satisfactory solutions, and only structural growth variation and connection weight learning can be carried out [23]. For structural growth evolutionary learning, the learning process will end only when a satisfactory solution is obtained. It is worth noting that the structure of the satisfactory solution network obtained at this time is often not satisfactory and optimal. For structural pruning evolutionary learning, when evolution stagnates and a satisfactory solution cannot be obtained, it indicates that the current population does not have the ability to obtain a satisfactory solution. It is determined that the best individual of the population before this pruning is the learning network with the smallest structural scale and the satisfactory optimal solution network.

## 4. Design of the Student Management System

### 4.1. System Requirements

From the perspective of system requirements analysis, as an application system to assist student management, this system is mainly aimed at colleges and departments with student management functions and relevant departments with students' comprehensive information needs. Since the management mode of students in our school is school work office ⟶ student management office of colleges and departments ⟶ teachers (mainly head teachers) and the head teachers are the direct managers of class students, some basic data of the student management information system need to be provided by the head teachers [24]. Ordinary teachers are responsible for the input and modification of students' grades. Therefore, the main objects of this system are school management staff, department student management staff, teachers, and students. The system requirements flow is shown in Figure 4.

### 4.2. System Function Analysis

#### 4.2.1. Function Analysis of the Student Status Subsystem

Through the statistical query of the data in the student files, various data statistical tables can be obtained. The student status management subsystem can manage all information changes of a student during school, such as student status change, punishment and reward management, and graduation management [25]. The data information in the subsystem is uniformly managed by the administrator, who has the authority to effectively manage the basic information, details, punishment, and graduation of students. The business flowchart of the student status subsystem is shown in Figure 5.

#### 4.2.2. Function Analysis of the Course Selection Subsystem

The course selection subsystem is a very important functional module in the college student management system. With reference to the curriculum of this semester offered by the college, all courses are listed. According to the actual situation of individuals and the arrangement of the college, courses are selected and confirmed to be submitted. If the data are legal, that is, the course selection is reasonable, the course selection application is submitted successfully and wait for the subsystem to process the course selection data accordingly. The business flowchart of the course selection subsystem is shown in Figure 6. Otherwise, students can reselect courses and repeat the above course selection process.

#### 4.2.3. Function Analysis of the Score Subsystem

At the end of the semester, teachers can enter the score management subsystem through their own teaching staff number and password and then enter all students' scores in their own teaching class through the score subsystem. Each teacher in the college may have multiple teaching courses or multiple classes, which can be distinguished by class number and course code [26]. Teachers can input students' course score information into the score database. The submission times of scores are specified as one time, but they can be modified many times. To modify scores, teachers need to fill in the modification application and get the approval of the academic affairs office of the school and then authorize teachers to modify scores through educational administration management personnel. The business flowchart of the score subsystem is shown in Figure 7.

#### 4.2.4. Function Analysis of the Curriculum Management Subsystem

At the beginning of each semester, students will choose courses, and administrators and teachers will set up courses, such as which courses need to be set up, which teacher will bring which course, as well as the place, time, and course information of the course. The management and maintenance of basic course information, the addition of new courses, the change of course credits, class hours, and elective/compulsory courses are the authorities of the administrator. Maintaining the information of teachers, courses, and classes, students choosing the courses they want to attend, viewing the selected credits and modifying their personal information, and teachers deciding the students to attend classes and giving students credits are the functional scopes of the course management, as shown in Figure 8, which is the functional analysis flowchart of the course management subsystem.

### 4.3. System UML Analysis

#### 4.3.1. Login Module Use Case Diagram

The use case diagram can well describe the role of the system. The following is the use case design diagram of the login system.

  Case name: login system
  Participants: administrators, teachers, and students
  Objective: to log into the student information management system
  Description: enter the user account and password, check the user name and corresponding password information stored in the database, and log in only after successful verification by the system. The system enables the user to enter the corresponding operation interface according to the user authority. If the account or password is entered incorrectly, a corresponding prompt will be generated, then exit the system and log in again. The use case diagram of login module is shown in Figure 9.

#### 4.3.2. Administrator Module Use Case Diagram

This system completes student information management, so the administrator in this system is mainly responsible for student information management, including adding, editing (deleting and modifying), and querying student information. The administrator manages student status information, student course information, and student achievement information. You can query, modify, and delete students' student status information, view students' selected courses, add and delete courses, view students' grades, and add and modify students' grades, as shown in Figure 10.

#### 4.3.3. Teacher Module Use Case Diagram

After logging into the system, teachers can manage all the information of their students, including basic information, reward and punishment information, achievement information, conduct evaluation information, course information, and so on. In addition, you can query the above data, as shown in Figure 11.

#### 4.3.4. Student Module Use Case Diagram

Student number is the only sign of students in school. After logging into the system with student number and password, students can query their own information, such as natural basic information, achievement information, reward information, punishment information, and course information, as shown in Figure 12.

### 4.4. System Function Module

It mainly includes the main management modules of student management, such as student information management, curriculum management, and performance management. The main functional modules completed by the system are shown in Figure 13.

System modification record refers to the modification of data records. First, after logging into the system, the user can check whether he has the permission to modify records. If he has the permission to modify records, it is allowed to query whether there are duplicate records in the database. For example, to modify a student's information in the system, first ask the database for the existence of the student through the student number. If so, the user is allowed to modify the data into the database and return to the successful modification interface. If it is found that the student number of the student does not exist in the system, the system fails to modify the record of the student information [27]. The process design of adding and modifying records in the system is shown in Figures 14 and 15.

System management is a module for managers to set permissions for users. Managers have the highest permissions and have all permissions on the system. The process design of system management is shown in Figure 16. First, after the login module, the system judges the user's permission according to the login record and assigns it to the corresponding operation of the user with the corresponding permission.

## 5. Effective Methods of Ideological and Political Work in the Internet+ Era

### 5.1. Existing Problems and Challenges of Ideological and Political Work in Colleges and Universities

#### 5.1.1. Traditional Problems and Challenges

(1) Thoughts and politics are dogmatic and difficult to adapt to new situations and changes in the new environment: at present, the method of ideological and political work has not completely got rid of the way of preaching. It is lack of innovation and difficulty to attract students. In the Internet+ era, students have been fully exposed to various external ideas and concepts, and there has been a trend of diversification. It is the responsibility of our ideological and political teachers in colleges and universities to guide college students to consciously maintain consistency in the main theme, promote positive energy, and identify those ideas that run counter to the main theme. However, if the working methods follow dogmatism and teach students through orders and preaching, it will be difficult to tell wonderful things. If students cannot listen, they cannot achieve the effect of education.

(2) Emphasis on academic performance, light ideological and political education, and lack of easiness to operate students' ideological and political assessment standards: in some cases, the ranking and measurement of student achievement in various awards are very rigorous and important. Students' ideological and political research is difficult; they do not pay attention to personal moral cultivation and do not strengthen ideological and political education and politics, and the operational measures of students' “ideological and political morality” are weak. As a result, some students only pay attention to professional learning and do not pay attention to personal ideological and political learning and moral cultivation.

#### 5.1.2. New Problems and Challenges in the Internet+ Era

(1) The ideological constraints of college students in the virtual world are weakened and easy to be affected by bad thoughts: the biggest difference between the Internet era and the non-Internet era is that in the latter, people's life circle is mainly acquaintances, and the behavior of college students mainly depends on the supervision of acquaintances, surrounding people and social public opinion and their inner beliefs. In the virtual world in the Internet+ era, on the one hand, without “acquaintances and people around,” everyone can be anonymous and unknown, which is easy to create the illusion that everyone does not know me. Therefore, it is difficult for acquaintances and public opinion to supervise. They mainly rely on their inner beliefs to supervise their behavior, which may lead to the weakening of college students' self-discipline. On the other hand, for college students, using the Internet has become a common way of life for college students. While the Internet brings all kinds of convenience, it also greatly affects their values, outlook on life, and world outlook. If students are influenced by bad thoughts, they may lead to all kinds of bad behaviors of some college students with poor self-discipline, which will harm all aspects. These new problems put forward new requirements for ideological and political education.

(2) In the real world, college students' face-to-face communication ability deteriorates: the life of contemporary college students is inseparable from the network. Many exchanges rely on various chat softwares. Some college students are easy to indulge in the virtual world of the network for a long time. Face-to-face communication between people is becoming less and less, which has become a common phenomenon among college students.

### 5.2. Effective Methods of Ideological and Political Work in the Internet+ Era

In view of the above problems and challenges, we must adopt scientific and effective new methods.

#### 5.2.1. Overcome Preaching and Use Students' Favorite Online Social Tools to Innovate Methods

“In order to function well in the thinking and politics of colleges and universities, we need to adapt to changing circumstances, progress over time, and innovate accordingly in the situation.” Now, college students get information from the Internet more than ever before. On the other hand, the network is designed and accelerated, so that college students will be able to know all the information in real time through the Internet. Some bad information will have an adverse effect on the thinking of college students, which requires us to pay close attention to the hot data on the Internet and the bad information that boys may encounter and respond and share in a timely manner [28]. On the other hand, college students rely on social networking every day. They should give full play to the role of the network, actively communicate with them, understand and find problems in time, and dredge and solve them.

#### 5.2.2. Constructing a New Measurement Method of Paying Equal Attention to Academic Achievement and Ideological and Political Work

Establish a comprehensive scientific standard or measurement to evaluate students' ideological and moral character. This measurement can not only quantify the quality of students in all aspects but also have the characteristics of easy operation. At the same time, the measurement of emotional and political and academic performance has been incorporated into the new measurement model, and the performance of the students has been extensively measured and researched on the purpose.

#### 5.2.3. Occupy the Dominance of Internet Discourse and Spread Positive Energy

In response to the negative impact that some of the ideas on the Internet can have on college students, on the one hand, educators and politicians need to pay close attention to collaborate in real time and spread the word more in purpose and work in the management of public opinion online through the use of social platforms frequently. On the other hand, we should also take the initiative to use social software to maintain regular and timely communication with students; understand the latest ideological trends, hobbies, and habits of students; pay attention to students' learning status; solve problems encountered in students' study and life; and care for students. By allowing students to participate in the production of small online videos with positive energy, online consultation, online interaction, smart classroom, and other ways, use the Internet to improve students' interest and enthusiasm in participating in ideological and political education, carry out rich and colorful educational publicity activities, and strive to be students' bosom friends and life mentors.

#### 5.2.4. Effective Use of Web-Based Technology and Management Platforms

Educators work through a web-based management platform, freeing them from many cumbersome approval processes and reducing waste of documents, paper, and other materials. At the same time, educators have more experience to devote to teaching and learning. In the past, reference materials, extra reading materials, and practice questions could be made available to students through online channels, that is, they could be easily accessed at any time and kept for a long time, reducing excessive waste of paper. For examinations, they can also be made available in an online format, increasing the speed of marking, reducing the amount of paper used for examinations, saving energy, and reducing carbon. On the other hand, students become aware of the importance of environmental protection during their studies and are implicitly involved in environmental activities.

## 6. Conclusion

Starting from the real needs of the system, this research is developed from software engineering concepts and network development and recognizes a way that is not only appropriate for nature but the current set of student data management also provides full play to the advantages of the net development framework and adheres to the development mode of web application systems, which are widely used. Based on the design and implementation, an example is used to test and analyze. First, through the analysis of the educational administration process of colleges and universities, the basic requirements for realizing the system are obtained. On this basis, the daily student information management business is analyzed, and the student information management system is designed according to the analysis results, which can help students, managers, and teachers manage information efficiently. The implementation of this website based on ASPNET technology environment has the advantages of openness, high performance, security, and low cost. Under the guidance of software engineering strategies, we use state-of-the-art technology to integrate system management and independence, giving full play to the quality of the network in data management and improving the operational efficiency of the system. At the same time, the system has mobility and versatility, which will help improve the performance of the students' information management system. As a case management system for undergraduate students, student management, especially the refinement of thought and politics, must be integrated with the background of the “Internet+” era and the frequent responses to the challenges brought by it. Develop a “Internet+” concept, effectively use the Internet platform to work on the management of thought and politics in colleges and universities, patiently learn, full use and develop state-of-the-art technology, hold on to ideas in online thought management and political education in a timely manner, and continue to expand the workplace to complete buildings college and university. To improve governance performance, ensure that the cultural and political administration in colleges and universities is in place, ensure that strongly promotes the achievement of cultural and economic excellence in colleges and universities, and ensure that these activities are always present in all race and demand from the state and community. Learn and apply the spirit of the National Conference on Ideological and Political Work in Colleges and Universities to highlight the importance of thought and politics in colleges and universities and introduce the guidance for the work of theoretical and political educators in colleges and universities. In light of the current state of the Internet+ era, this study presents the uniqueness and importance of the ideological and political work in colleges and universities of medicine, examines issues and problems encountered by thought and politics in colleges and universities in the Internet+ era, and adds procedures to address issues and problems.

## Figures and Tables

**Figure 1:** Student ideological and political management model.

**Figure 2:** EPNN evolutionary learning system.

**Figure 3:** Evolutionary algorithm flow.

**Figure 4:** System analysis flowchart.

**Figure 5:** Student status business flowchart.

**Figure 6:** Flowchart of course selection.

**Figure 7:** Performance management business flowchart.

**Figure 8:** Flowchart of the course arrangement.

**Figure 9:** Login module use case diagram.

**Figure 10:** Admin module use case diagram.

**Figure 11:** Use case diagram of teacher management module.

**Figure 12:** Use case diagram of student management module.

**Figure 13:** System function module diagram.

**Figure 14:** Flowchart of adding record module.

**Figure 15:** Flowchart of modification record module.

**Figure 16:** Flowchart of system management module.

## Data Availability

The dataset used to support the findings of this study is available from the corresponding author upon request.
